# Association of brain natriuretic peptide gene polymorphisms with chronic obstructive pulmonary disease complicated with pulmonary hypertension and its mechanism

**DOI:** 10.1042/BSR20180905

**Published:** 2018-10-02

**Authors:** Guangjun Jin, Zhu Chen, Jiancheng Zhang, Jia Song, Jun Shi, Bingzhi Zhou

**Affiliations:** 1 Department of Emergency, the Second Affiliated Hospital of Zhejiang Chinese Medical University, 318 Chaowang Road, Hangzhou, Zhejiang, China; 2 Department of Clinical Laboratory, Ningbo No. 2 Hospital, No. 41 Northwest Street, Haishu District, Ningbo City, Zhejiang Province, China

**Keywords:** Brain natriuretic peptide, Chronic obstructive pulmonary disease, Pulmonary hypertension, Single nucleotide polymorphism

## Abstract

**Objective:** To examine the association between brain natriuretic peptide (BNP) gene single nucleotide polymorphisms (SNPs) and chronic obstructive pulmonary disease (COPD) and COPD with pulmonary hypertension (PH) and to analyze its mechanism. **Methods:** The genotypes of *BNP* at the rs198389, rs6668352, and rs198388 loci in 339 patients with COPD (205 in the COPD/PH^−^ group and 134 in the COPD/PH^+^ group) and 125 healthy subjects were detected by PCR/Sanger sequencing. The serum levels of BNP, fibrinogen (Fbg), and Apelin were measured in all subjects by ELISA. **Results:** The *BNP* rs198389 locus G allele, rs6668352 locus A allele, and 198388 locus T allele were high risk factors for COPD (*P*<0.001). Logistics regression analysis showed that *BNP* rs198389 locus G allele, rs6668352 locus A allele, and rs198388 locus T allele were high risk factors for PH in COPD patients (all *P*<0.001). The levels of the serum BNP and Fbg protein in the control group, COPD/PH^−^ group, and COPD/PH^+^ group increased successively, and the expression levels of Apelin protein decreased successively (all *P*<0.001). The BNP and Fbg protein levels in the wild-type, heterozygote, and mutant homozygote in *BNP* rs198389, rs6668352, and rs198388 loci increased successively, and the serum Apelin protein levels decreased successively (all *P*<0.001). **Conclusion:** The polymorphisms of *BNP* at the rs198389, rs6668352, and rs198388 loci are associated with the occurrence of COPD and COPD with PH, and the occurrence may be related to the abnormal expression level of BNP, Fbg, and Apelin protein in the serum.

Chronic obstructive pulmonary disease (COPD) is a common chronic disease, and its incidence has gradually increased recently [1]. Pulmonary hypertension (PH) is a common complication of COPD, which seriously affects the prognosis and quality of life of patients [2]. Previous studies show that the occurrence of COPD is related to factors such as the living environment, air quality, smoking history, and genetic factors [3]. There are few studies on the correlation between COPD and COPD with PH and genetic factors.

Brain natriuretic peptide (BNP) is a functional peptide synthesized by cardiomyocytes, and its function is mainly to regulate the physiological balance of blood pressure and blood flow [4]. Studies show that BNP plays an important role in the diagnosis of heart failure, hypertension, and cardiopulmonary diseases [5,6]. For example, Chen et al. [7] showed that N-terminal hormone BNP (NT-proBNP) has a certain value in the rapid diagnosis of patients requiring hospitalization for AECOPD. At present, many single nucleotide polymorphism (SNP) loci of the BNP gene are associated with hypertension and chronic heart failure. A study by Zhang et al. [8] showed that the BNP gene SNP loci rs198389 and rs198388 are associated with the genetic susceptibility to congenital heart disease. Poreba et al. [9] showed that the SNP at the rs198389 site of the BNP gene is associated with the development of atherosclerotic lesions in the renal artery. In addition, Fox et al. [10] studies showed that the rs198389, rs6668352, and rs198388 SNP sites of the BNP gene were associated with ventricular dysfunction (VnD) after primary coronary bypass surgery. However, there are few studies on the association between gene polymorphisms of the BNP genes rs198389, rs6668352, and rs198388 and the occurrences of COPD and COPD with PH. The associations between SNPs in the BNP genes, including rs198389, rs6668352, and rs198388, and COPD and COPD with PH were analyzed. This article focuses on this issue. Apelin is a small molecule polypeptide, and studies show that Apelin can be used as an effective indicator of COPD associated with a diagnosis of PH [11]. Fibrinogen (Fbg) is a protein that is present in plasma. The level of plasma Fbg is positively related to the severity of COPD and thus can be used to reflect the severity of COPD [12].

## Methods

### General information

A total of 339 patients with COPD from August 2014 to August 2017 were enrolled in the present study; according to whether they were complicated with PH, they were subdivided into a COPD/PH^−^ group (205 cases) and a COPD/PH^+^ group (134 cases). The diagnostic criteria of COPD was based on the Global Initiative for Chronic Obstructive Lung Disease (GOLD) [] {13}. The diagnosis of PH is based on the 2015 guideline for the diagnosis and treatment of PH in ESC/ERS [14], excluding patients with bronchial asthma, tuberculosis, lung cancer, bronchiectasis, interstitial fibrosis, and other respiratory diseases as well as patients with hypertension, malignancy, and connective tissue disease. A total of 125 healthy subjects [forced expiratory volume in one second as a percentage of the predicted (FEV_1_%) ≥80% and forced expiratory volume in one second/forced vital capacity (FEV_1_/FVC) ≥70%] without chronic bronchitis and emphysema were enrolled as the control group. The study was approved by our medical ethics committee, and all the participants signed an informed consent (approval number: 201407013).

### Clinical data collection

Clinical data from all subjects were collected, including their age, sex, course of disease, body mass index (BMI), and smoking index (number of cigarettes per year). The blood gas parameters of the COPD/PH patients were measured with a blood gas analyzer, and the lung function of the subjects was measured with a *V*_max_ pulmonary function meter, including the FEV_1_ as a percentage of the predicted value, the FVC, the arterial partial pressure PaO_2_, and the arterial carbon dioxide partial pressure PaCO_2_.

### Methods of collecting and treating blood

From all subjects, we collected 5 ml of fasting venous blood, of which 3 ml was used to separate the serum after coagulation. The expressions of the BNP (Ek-Bioscience, CAT#: EK-H11285), Fbg (Elabscience, CAT#: E-EL-M0498c), and Apelin (Elabscience, CAT#: E-EL-R2413c) proteins in the serum were detected by ELISA. After anticoagulation by adding EDTA-K2, the remaining 2 ml of blood was subjected to the QIAamp DNA Blood Mini Kit (Qiagen, 51106, German) to extract the genomic DNA. All experimental operations were performed strictly in accordance with the kit instructions.

### Genotyping of the BNP gene rs198389, rs6668352, and rs198388 loci

Using the extracted gDNA as a template, the target DNA fragment was amplified by PCR. The amplified primers at each locus and the reaction system and conditions of the PCR amplification reaction are shown in Table 1. After PCR, the PCR product was purified by a DNA Gel Extraction Kit (Beyotime, CAT#:0056), and the sequence of the target DNA was detected by Sanger sequencing. The results are shown in Figure 1.

**Figure 1:** The sequencing results of the PCR product of the BNP gene A, B, and C were wild-type (AA-type), heterozygous (AG-type), and homozygous mutants (GG-type) of the BNP gene rs198389 locus, respectively. D, E, and F were wild-type (GG type), heterozygous (GA type), and homozygous mutants (AA type) of the BNP gene rs6668352 locus, respectively. G, H, and I were wild-type (CC type), heterozygous (CT type), and mutant homozygous (TT type) of BNP gene rs198388 locus, respectively.

**Table 1:** PCR amplification information of the BNP gene rs198389, rs6668352, and rs198388 loci

SNP loci	Primer sequence (5′ to 3′)	PCR mix	PCR procedure
rs198389	Forward primer: AGACACAGACAAGTCCCCGT; Reverse primer: GAAAGCGCCAACCTAGGACA	ddH_2_O: 13.8 μl; 10× PCR buffer: 2 μl; 10 mM dNTP mix: 1 μl; Primer Forward: 1 μl; Primer Reverse: 1 μl; Taq DNA Polymerase: 0.25 μl; genomic DNA: 1 μl	95°C, 5 min (94°C, 45 s; 58°C, 45 s; 72°C, 30 s) 30 cycles; 72°C, 10 min
rs6668352	Forward primer: TGTCACTCACTGGGTACAGC; Reverse primer: ACCTGCGAAGGAGCCAAATG		
rs198388	Forward primer: TTCTCCCAAGTGCCTCAAGT; Reverse primer: AGGTAGCAGGCTTTCTTTTCT		

### Statistical analysis

The statistical analysis of the data was performed using SPSS 20.0 software (SPSS Inc., Chicago). The continuous and non-parametric data are represented by (±s), and the categorical variables are represented by [*n*(%)]. The Pearson chi-square test was used to compare the classification variables. The average values of the continuous variables of the normal distribution were compared by one-way analysis of variance (ANOVA). The Mann–Whitney *U* test was used to compare the skewed distributions of the continuous variables. A non-parametric statistical analysis between the two groups was performed using a *t-*test. The *χ*^2^ test was used to detect whether the genotype frequencies were consistent with the Hardy–Weinberg equilibrium. The odds ratio (OR) and the 95% confidence interval (CI) were used to analyze the correlations between the genotypes and COPD and COPD with PH. A multivariate logistic regression analysis was used to correct the factors such as the age, gender, BMI, and smoking index. *P*<0.05 indicated that the difference was statistically significant.

## Results

### Comparison of the clinical parameters

The clinical parameters of the subjects in the control group, COPD/PH^−^ group, and COPD/PH^+^ group are shown in Table 2. There were no significant differences in the clinical parameters, including the age, gender, BMI, and smoking index, amongst the three groups (*P*>0.05). There was no significant difference in the course of disease between the COPD/PH^−^ group and the COPD/PH^+^ group (*P*>0.05). The PaCO_2_ of the subjects in the control group, COPD/PH^−^ group, and COPD/PH^+^ group increased successively, while the FEV_1_/predicted value, FEV_1_/FVC, FVC, and PaO_2_ decreased successively, and the differences were statistically significant (*P*<0.05).

**Table 2:** Comparison of the general clinical data amongst the three groups

Index	Control group (*n*=125)	COPD/PH^−^ group (*n*=205)	COPD/PH^+^ group (*n*=134)	*P*-value
Age (years)	63.8 ± 5.3 (49, 76)	64.2 ± 4.8 (45, 77)	64.5 ± 5.2 (45, 77)	0.597
Gender [male, *n* (%)]	68 (54.4%)	112 (54.6%)	81 (60.4%)	0.291
Course (years)	–	16.1 ± 5.8 (2, 27)	16.4 ± 5.5 (5, 27)	0.635
BMI (kg/m^2^)	22.8 ± 2.4 (18.9, 26.1)	22.5 ± 2.4 (16.7, 27.5)	22.4 ± 2.5 (17.8, 27.3)	0.490
Smoking (pack/year)	31.6 ± 3.7 (24, 38)	32.4 ± 4.1 (23, 39)	32.0 ± 4.1 (23, 39)	0.221
FEV_1_/predicted value (%)	80.8 ± 12.4 (53, 96)	43.5 ± 4.7 (32, 63)	43.6 ± 5.1 (30, 65)	<0.001
FEV_1_/FVC (%)	73.5 ± 13.4 (56, 86)	55.6 ± 11.4 (43, 72)	53.5 ± 12.1 (40, 76)	<0.001
FVC (%)	82.1 ± 20.4 (65, 97)	49.2 ± 17.5 (32, 61)	40.5 ± 16.7 (26, 58)	<0.001
PaO_2_ (mmHg)	88.0 ± 6.1 (76.5, 98.5)	62.6 ± 8.3 (54.2, 73.6)	54.5 ± 4.0 (51.2, 59.7)	<0.001
PaCO_2_ (mmHg)	44.2 ± 4.2 (36.8, 52.3)	60.8 ± 7.6 (51.2, 66.7)	66.4 ± 7.6 (58.4, 72.4)	<0.001
SpO_2_ decreased by 3% during exercise	27 (21.6%)	123 (48.3%)	105 (85.1%)	<0.001
D-dimer (μg/l)	307.5 ± 205.4 (102.5, 495.4)	498.4 ± 207.6 (208.6, 603.7)	651.7 ± 325.6 (422.8, 982.7)	<0.001
6MWT/m	413.8 ± 45.3 (375.8, 462.1)	312.6 ± 39.8 (264.4, 345.7)	250.5 ± 36.5 (214.5, 295.6)	<0.001
DLCO/%	88.5 ± 12.3 (70.5, 95.8)	56.5 ± 7.8 (44.8, 72.3)	55.7 ± 7.6 (45.4, 69.8)	<0.001
mPAP/mmHg	20.1 ± 2.5 (17.9, 23.1)	23.5 ± 2.7 (19.2, 24.9)	36.7 ± 5.7 (31.6, 43.8)	<0.001
Pulmonary vascular resistance (WU)	1.1 ± 0.3 (0.9, 1.4)	2.4 ± 0.5 (2.2, 2.7)	4.6 ± 0.7 (4.2, 4.9)	<0.001
Cardiac output (l/min)	5.9 ± 1.1 (5.1, 6.8)	6.5 ± 1.2 (5.7, 7.6)	6.1 ± 1.4 (5.5, 7.7)	0.764
Cardiac index (l/min/m^2^)	2.5 ± 0.9 (2.0, 3.9)	3.7 ± 1.4 (2.9, 4.9)	3.4 ± 1.6 (2.7, 5.3)	0.217
GFR (ml/min × 1.73 m^2^)	87.6 ± 4.1 (48.4, 102.3)	78.5 ± 3.6 (45.5, 99.6)	62.5 ± 3.1 (37.1, 81.4)	0.007
RBF (ml/min × 1.73 m^2^)	1054.6 ± 65.2 (706.9, 135.4)	851.2 ± 42.3 (760.1, 991.3)	653.8 ± 33.9 (583.4, 701.4)	<0.001

FVC (minimum, maximum). Abbreviations: GFR, glomerular filtration rate; 6MWT, 6 min walking tests; RBF, renal blood flow.

### The correlations between the SNPs of the BNP gene, including the rs198389, rs6668352, and rs198388 loci, and COPD

The genotype distributions of the BNP gene SNP loci rs198389, rs6668352, and rs198388 of the subjects in the three groups are shown in Table 3. The percentage of the rs198389 site homozygous mutation of the BNP gene in the COPD group was significantly higher than that of the control group (adjusted OR = 1.265, 95% CI = 1.100–1.407, *P*=0.001), and the risk of COPD in the G allele carriers increased significantly (adjusted OR = 1.165, 95% CI = 1.076–1.254, *P*<0.001). The percentage of the rs6668352 site homozygous mutation of the BNP gene in the COPD group was significantly higher than that in the control group (adjusted OR = 1.327, 95% CI = 1.158–1.463, *P*<0.001), and the risk of COPD in the A allele carriers increased significantly (adjusted OR = 1.199, 95% CI = 1.108–1.288, *P*<0.001). The ratio of the rs198388 site homozygous mutation of the BNP gene in the COPD group was significantly higher than that of the control group (adjusted OR = 1.261, 95% CI = 1.091–1.396, *P* = 0.002), and the risk of COPD in the T allele carriers increased significantly (adjusted OR = 1.145, 95% CI = 1.055–1.232, *P*<0.001).

**Table 3:** Genotypic distributions of the rs198389, rs6668352, and rs198388 loci in the BNP gene in the control group and the COPD group

SNPs	Control group (*n*=125)	COPD group (*n*=339)	*P*-value	OR (95% CI)	*P-*value*	OR* (95% CI)
rs198389 genotype						
AA	69 (55.2%)	141 (41.6%)	1.00			
AG	40 (32.0%)	108 (31.9%)	0.238	1.321 (0.811–2.157)	0.287	1.087 (0.937–1.247)
GG	16 (12.8%)	90 (26.5%)	0.005	2.753 (1.450–5.282)	0.001	1.265 (1.100–1.407)
Allele						
A	178 (71.2%)	390 (57.5%)	1.00			
G	72 (28.8%)	288 (42.5%)	<0.001	1.826 (1.319–2.529)	<0.001	1.165 (1.076–1.254)
rs6668352 genotype						
GG	71 (56.8%)	137 (40.4%)	1.00			
GA	41 (32.8%)	112 (33.0%)	0.136	1.416 (0.873–2.299)	0.169	1.111 (0.958–1.276)
AA	13 (10.4%)	90 (26.5%)	<0.001	3.588 (1.804–7.248)	<0.001	1.327 (1.158–1.463)
Allele						
G	183 (73.2%)	386 (56.9%)	1.00			
A	67 (26.8%)	292 (43.1%)	<0.001	2.066 (1.485–2.878)	<0.001	1.199 (1.108–1.288)
rs198388 genotype						
CC	68 (54.4%)	147 (43.4%)	1.00			
CT	45 (36.0%)	117 (34.5%)	0.419	1.203 (0.750–1.931)	0.488	1.056 (0.916–1.208)
TT	12 (9.6%)	75 (22.1%)	0.001	2.891 (1.414–6.017)	0.002	1.261 (1.091–1.396)
Allele						
C	181 (72.4%)	411 (60.6%)	1.00			
T	69 (27.6%)	267 (39.4%)	<0.001	1.704 (1.226–2.371)	0.001	1.145 (1.055–1.232)

* Corrected according to age, sex, BMI, smoking index, and other clinical parameters.

### The correlation between the rs198389, rs6668352, and rs198388 loci SNP in the BNP gene and COPD complicated with PH

The genotypic distributions of the rs198389, rs6668352, and rs198388 loci in the BNP gene in the COPD/PH^−^ and COPD/PH^+^ groups are shown in Table 4. The proportion of homozygous mutations in the rs198389, rs6668352, and rs198388 loci in the COPD/PH^+^ group was significantly higher than in the COPD/PH^−^ group (*P*<0.001). The results of the logistic regression analysis showed that the G allele at the rs198389 locus, the A allele at the rs6668352 locus, and the T allele at the rs198388 locus of *BNP* were high risk factors for the COPD patients complicated with PH (adjusted OR = 2.426, 95% CI = 1.992–2.955, *P*<0.001; adjusted OR = 2.257, 95% CI = 1.853–2.747, *P*<0.001; and adjusted OR = 1.842, 95% CI = 1.524–2.219, *P*<0.001, respectively).

**Table 4:** Genotypic distributions of the rs198389, rs6668352, and rs198388 loci in the *BNP* gene in the COPD/PH^−^ group and COPD/PH^+^ group

SNPs	COPD/PH^−^ group (*n*=205)	COPD/PH^+^ group (*n*=134)	*P*-value	OR (95% CI)	*P*-value*	OR* (95% CI)
rs198389 genotype						
AA	105 (51.2%)	36 (26.9%)	1.00			
AG	84 (41.0%)	24 (17.9%)	0.545	0.833 (0.442–1.566)	0.649	0.870 (0.532–1.403)
GG	16 (7.8%)	74 (55.2%)	<0.001	13.490 (6.661–27.666)	<0.001	3.220 (2.444–4.094)
Allele						
A	294 (71.7%)	96 (35.8%)	1.00			
G	116 (28.3%)	172 (64.2%)	<0.001	4.541 (3.223–6.403)	<0.001	2.426 (1.992–2.955)
rs6668352 genotype						
GG	106 (51.7%)	31 (23.1%)	1.00			
GA	75 (36.6%)	37 (27.6%)	0.067	1.687 (0.927–3.074)	0.091	1.460 (0.946–2.258)
AA	24 (11.7%)	66 (49.3%)	<0.001	9.403 (4.871–18.302)	<0.001	3.241 (2.342–4.426)
Allele						
G	287 (70.0%)	99 (36.9%)		1.00		
A	123 (30.0%)	169 (63.1%)	<0.001	3.983 (2.838–5.594)	<0.001	2.257 (1.853–2.747)
rs198388 genotype						
CC	100 (48.8%)	47 (35.1%)	1.00			
CT	89 (43.4%)	28 (20.9%)	0.150	0.669 (0.373–1.199)	0.193	0.748 (0.485–1.139)
TT	16 (7.8%)	59 (44.0%)	<0.001	7.846 (3.908–15.928)	<0.001	2.460 (1.890–3.063)
Allele						
C	289 (70.5%)	122 (45.5%)	1.00			
T	121 (29.5%)	146 (54.5%)	<0.001	2.858 (2.048–3.991)	<0.001	1.842 (1.524–2.219)

* Corrected according to age, sex, BMI, smoking index, and other clinical parameters.

### Analysis of serum BNP, Fbg, and Apelin protein expression

The results of the ELISA detection of serum BNP, Fbg, and Apelin protein expression in the subjects are shown in Table 5. The expressions of BNP and Fbg protein in the control group, COPD/PH^−^ group and COPD/PH^+^ group increased sequentially (*P*<0.001), while the expression levels of the Apelin protein in the control group, COPD/PH^−^ group and COPD/PH ^+^ group decreased sequentially (*P*<0.001).

**Table 5:** Comparison of the plasma BNP, Fbg, and Apelin content in the three groups ($\bar{\text{x}}$ ± s)

Plasma parameters	Control group (*n*=125)	COPD/PH^−^ group (*n*=205)	COPD/PH^+^ group (*n*=134)	*P*-value
BNP (ng/l)	28.1 ± 9.8	158.6 ± 23.0	220.2 ± 18.9	<0.001
Fbg (g/l)	2.5 ± 0.5	4.2 ± 0.5	5.4 ± 0.8	<0.001
Apelin (ng/l)	90.5 ± 8.4	43.9 ± 4.6	29.4 ± 6.2	<0.001

### The correlation between the rs198389, rs6668352, and rs198388 loci SNPs in the BNP gene and serum protein content of BNP, Fbg, and Apelin

The BNP, Fbg, and Apelin protein expressions in the subjects for each genotype of the *BNP* gene for the loci rs198389, rs6668352, and rs198388 are shown in Figure 2. According to the results, the content of BNP and Fbg protein in the serum of the heterozygote and mutant homozygote at the *BNP* gene rs198389, rs6668352, rs198388 loci increased successively, while the content of serum Apelin protein decreased successively (*P*<0.001).

**Figure 2:** Comparison of plasma BNP, Fbg, and Apelin protein content in subjects with each genotype of BNP gene rs198389, rs6668352, and rs198388 loci ***P<0.001.

### Correlation between BNP gene rs198389, rs6668352, rs198388 locus SNP and serum IL-6, IL-8 levels

The levels of IL-6 and IL-8 in serum were detected by ELISA, as shown in Figure 3. The results showed that the serum levels of IL-6 and IL-8 in wild-type, heterozygote, and homozygote of BNP gene rs198389, rs6668352, and rs198388 were increased in turn (*P*<0.05).

**Figure 3:** Comparison of plasma IL-6, IL-8 expression levels in subjects with genotypes of the BNP gene rs198389, rs6668352, and rs198388 loci ***P<0.001; **P<0.01, *P<0.05.

### Data availability statement

All data generated during and/or analyzed during the current study are available from the corresponding author upon reasonable request.

## Discussion

PH often accompanies patients with advanced COPD; the pulmonary vascular endothelial cells and smooth muscle cells in these patients are abnormal, and they have pulmonary vascular remodeling and right heart failure, which can cause death in severe cases [15]. The occurrence of COPD is associated with lung airway inflammation in patients, and airway restriction is also one of the clinical features of COPD [16]. Fbg is a blood coagulation factor and one of the lung airway inflammation markers [17]. Studies show that serum Fbg content reflects the severity of COPD, and in patients with exacerbated COPD, it is significantly higher [18]. The results of the present study showed that the serum Fbg content in COPD/PH^+^ patients was significantly higher than in COPD/PH^−^ patients [(5.4±0.8) g/l vs. (4.2±0.5) g/l], which was in agreement with the results by Ilisie et al. [18]. Furthermore, a comparison of the expression of serum Fbg protein in the subjects with different genotypes showed that the Fbg protein content of the wild types of the BNP gene rs198389, rs6668352, and rs198388 loci is lower than heterozygotes, and that of heterozygotes is lower than that of mutant homozygotes (all *P*<0.05), indicating that mutations in the rs198389, rs6668352, and rs198388 loci of the BNP gene lead to an increased expression of Fbg in the serum and increased lung airway inflammation in the mutant gene carriers. We speculated that this may be one of the causes of PH in the patients with COPD.

Apelin is a small molecule polypeptide that is an endogenous ligand for the orphan G protein-coupled receptor APJ. It has many biological effects, such as lowering blood pressure, enhancing myocardial contractility, regulating immunity, and regulating water and salt balances [19–21]. A study showed that Apelin could reduce myocardial damage in the PH rat model induced by monocrotaline and improve their right ventricle function [22]. Clinical studies show that the serum levels of Apelin in patients with PH are reduced, and an exogenous supplementation of it improves the clinical symptoms of PH to a certain extent and increases the cardiac output of patients with PH [23]. Recently, a serum Apelin test was used as a very important way to diagnose the severity of PH [24]. The results of the present study showed that the serum Apelin in patients with COPD is significantly lower than that in the control group, and the serum Apelin in the COPD/PH^+^ group is lower than that in the COPD/PH^−^ group, indicating that, with the worsening of COPD in patients, the expression of Apelin in the serum gradually decreases, which is consistent with the findings by Andersen et al. In addition, the present study analyzed the correlation between BNP gene SNPs and serum Apelin expression levels. The results showed that the content of Apelin protein in the serum of the heterozygote and mutant homozygote at the BNP gene rs198389, rs6668352, and rs198388 loci decreased successively. In addition, the present study analyzed the correlation between the BNP gene SNPs and the serum Apelin content, which showed that the serum Apelin protein in the wild types of the BNP gene rs198389, rs6668352, and rs198388 loci is higher than that of heterozygotes, and that of heterozygotes is higher than that of mutant homozygotes (all *P*<0.05), indicating that mutations at the rs198389, rs6668352, and rs198388 sites of *BNP* resulted in a decrease in serum Apelin protein, which may be one of the causes of the exacerbations of COPD, and thus, it might be used as a potential therapeutic target for COPD with PH.

BNP is located on human chromosome 1, which contains three exons and two introns encoding the BNP prohormone precursor [25]. The BNP prohormone precursor is synthesized in cardiac myocytes and is then processed under shear stress and secreted into the plasma to regulate blood pressure and blood flow to maintain homeostasis [26]. Studies show that plasma BNP levels may be associated with postoperative low cardiac output syndrome in children with congenital heart disease. Approximately 90% of PH patients who undergo congenital heart disease surgery have a preoperative plasma BNP higher than 125.5 pg/ml, leading to an increased risk of low cardiac output syndrome [27]. Studies show that an elevated BNP level is associated with heart failure and that the detection of the BNP content is expected to be used for clinical heart failure screening [28]. Left ventricular systolic dysfunction (LVSD) and cardiac decompensation are usually accompanied by AECOPD, and studies have shown that NT-proBNP can be used as a diagnostic marker for LVSD in acute exacerbation of COPD [29]. The results of the present study showed that the serum BNP level in patients with COPD was significantly higher than that in the control group. With the exacerbation of COPD patients, the serum BNP expression level gradually increased, which was consistent with the results by Inoue et al. [30]. At the same time, the present study also analyzed the correlation between the BNP gene SNPs and serum BNP expression levels, which showed that the content of the BNP protein in the serum of the wild types at the BNP gene rs198389, rs6668352, and rs198388 loci is lower than that of heterozygotes and that of heterozygotes is lower than that of mutant homozygotes (all *P*<0.001), indicating that mutations in the BNP gene at the rs198389, rs6668352, and rs198388 SNPs resulted in the elevation of BNP and might be one of the causes of COPD and COPD with PH.

In addition, we also analyzed the correlation between the polymorphisms of the *BNP* rs198389, rs6668352, rs198388 loci and the levels of IL-6 and IL-8 in serum. The results showed that the levels of IL-6 and IL-8 in the *BNP* rs198389, rs6668352, and rs198388 mutants were higher than those in the wild type. COPD usually activates inflammatory cells to release inflammatory mediators, such as IL-6 and IL-8, and IL-6 can induce inflammation by secreting cytokines such as IgG, IgA, and IgE through promoting cell maturation [31]. IL-8 is an endogenous chemokine of inflammatory cells, whose main role is to chemotactic neutrophils, elevate the intracellular concentration of Ca^2+^, resulting in increased histamine release in peripheral blood and trigger inflammatory reaction [32]. The elevated levels of IL-6 and IL-8 in the serum of subjects with BNP gene rs198389, rs6668352, and rs198388 mutations in the present study indicate that these SNPs are involved in the development of inflammatory response and may contribute to COPD. Ghobadi et al. [33] showed that the levels of serum IL-6 and pro-BNP increased with the severity of COPD, and the results were consistent with the results of the present study.

The present study also had some limitations. First, the present study did not analyze the impacts of different ethnic groups on gene polymorphisms at the rs198389, rs6668352, and rs198388 loci of the BNP gene and did not distinguish amongst different ethnic groups when enrolling the subjects. Second, in order to understand the effect of the BNP polymorphisms on the natriuretic peptide pathway, other natriuretic peptides, including atrial natriuretic peptide and C-type natriuretic peptide, should also be included in the study.

## Conclusion

Gene polymorphisms of the BNP gene, including rs198389, rs6668352, and rs198388, were associated with COPD and COPD with PH. Mutant individuals were more susceptible to COPD and prone to PH. The mechanism may be related to the high expression of BNP and Fbg protein in the serum and the abnormally low expression of the Apelin protein.

## Abbreviations

AECOPD: acute exacerbation of chronic obstructive pulmonary disease
BMI: body mass index
BNP: brain natriuretic peptide
CI: confidence interval
COPD: chronic obstructive pulmonary disease
Fbg: fibrinogen
FEV_1_: forced expiratory volume in one second
FVC: forced vital capacity
IgA/IgE/IgG: immunoglobulins A, E and G
IL: Interleukin
LVSD: left ventricular systolic dysfunction
NT-proBNP: N-terminal hormone brain natriuretic peptide
OR: odds ratio
PH: pulmonary hypertension
SNP: single nucleotide polymorphism
